The article "Identified PAH V230A and PAH V230I mutations in a family with diverse clinical presentations" was published in 2024. Journal: Clin Case Rep.

# Identified PAH V230A and PAH V230I mutations in a family with diverse clinical presentations

**DOI:** 10.1002/ccr3.8598

**Published:** 2024-03-12

**Authors:** Faeze Khaghani, Peyman Eshraghi, Tayebeh Hamzehloei

**Affiliations:** ^1^ Department of Pharmaceutical Biotechnology, School of Pharmacy Guilan University of Medical Sciences Rasht Iran; ^2^ Department of Human Genetics, School of Medicine Mashhad University of Medical Sciences Mashhad Iran; ^3^ Department of Pediatric and Endocrinology, School of Medicine Mashhad University of Medical Sciences Mashhad Iran; ^4^ Metabolic Syndrome Research Centre Mashhad University of Medical Sciences Mashhad Iran

**Keywords:** endocrinology and metabolic disorders, genetics and genomics, health informatics, pathology and laboratory medicine, pediatrics and adolescent medicine

## Abstract

Phenylketonuria (PKU) is a hereditary disorder caused by phenylalanine hydroxylase enzyme (PAH) defects that might cause severe brain damage. The current main treatment, dietary management, can prevent the symptoms if commenced early. However, it has side effects if used for a long time. Additionally, some patients with mild hyperphenylalaninemia (mHPA), who has serum phenylalanine levels <360 μmol/L, do not require treatment. Since the correlation between genotype and metabolic phenotype has been demonstrated earlier, genotype‐based detection of patients who do not need treatment might help with genetic counseling and choosing the most appropriate treatment option. In this study, we report an asymptomatic adult with mHPA who had never taken any medical intervention to control or lower her serum phenylalanine level (Phe). She had 179 μmol/L serum phenylalanine level and carried p.[V230A];[V230I] genotype. Her child was affected with phenylketonuria and had p.[V230A];[V230A] genotype. Both pathogenic variants detected in the asymptomatic adult with mHPA were computationally analyzed to assess their pathogenicity and the p.V230I pathogenic variant was demonstrated to be responsible for the mHPA phenotype in the asymptomatic adult detected in this study. The findings in this study could contribute to genetic counseling and treatment for families and individuals with p.[V2030I];[V230A] genotype.

## 1 INTRODUCTION

Phenylketonuria (PKU; OMIM#261600) is a hereditary disorder resulting from defects in phenylalanine hydroxylase enzyme (PAH, EC 1.14.16.1), following pathogenic variants within the *PAH* gene. The *PAH* gene, which spans 13 exons, is located on the 12q22‐q24.1 chromosome and encodes the *PAH* enzyme, which is in charge of converting phenylalanine (Phe) to tyrosine (Tyr).^1^ PAH deficiency results in the accumulation of Phe, which has many adverse effects that are still not fully understood.^2^

The article "Identified PAH V230A and PAH V230I mutations in a family with diverse clinical presentations" was published in 2024. Journal: Clin Case Rep.

Following a low‐Phe diet and trying a Phe‐lowering medicine are current treatment options that aim to lower Phe concentration in blood.^3^, ^4^ In fact, dietary treatment can prevent the mentioned complications if started immediately after birth. Despite the benefits of dietary management, a PKU diet that is followed for an extended period of time is linked to vitamin and/or mineral deficiencies^5^, ^6^, ^7^ as well as an enhanced risk of low bone density.^8^ Treatment for life is still recommended for any patient with PKU, despite the fact that diet management is associated with a significant patient burden.^8^

The last US and European guidelines recommend initiating treatment at a Phe level greater than 360 μmol/L,^1^ and Phe level should be kept below 360 μmol/L for children and pregnant women.^1^ Nevertheless, the US guidelines also suggest serum Phe levels should be maintained <360 μmol/L in individuals who are in their teenage years or older, based on the idea that the closer the Phe level is to physiological the better the outcome.^1^ However, it is suggested to be retained <600 μmol/L in individuals who are over 12 years old or older by European guidelines.^1^

The serum Phe concentration before treatment is also the main basis of the classification of phenotype,^9^ which is mainly categorized into three groups: typical PKU, mild PKU, and mild hyperphenylalaninemia (mHPA, mild HPA, or Benign HPA).^9^ The mHPA is further divided as HPA with a pretreatment Phe concentration of 120–360 μmol/L or 360–600 μmol/L, although pediatric cases were reported who showed an unexpected progression to >360 μmol/L category at follow‐up.^10^

These phenotypes result mainly from different mutations within the PAH gene. Mild HPA is a condition caused by hypomorphic variants which result in low but adequate levels of the enzyme.^11^ Therefore, it is not considered serious and does not have a definitive clinical significance.^11^ This decreased activity keeps the Phe level low enough to prevent serious neurodevelopmental disorders. Because an association between genotypes and in vitro residual enzyme activity has been shown for a large number of PAH variants,^12^ phenotype prediction based on genotype might be clinically beneficial, especially for genetic counseling of patients' families or in case treatment recommendations are unclear.^13^ Recognizing patients who might present mHPA phenotype and who do not need lifelong diet and supplementation might contribute to genetic counseling, treatment, and avoiding dietary restriction problems.

In this essay, a consanguineous family with a PKU‐affected child and her parent (an asymptomatic adult with mHPA [detected during the study], and an asymptomatic subject) was analyzed for PAH mutations. The genotype of the normal adult with mHPA and both mutations were separately computationally investigated to find the reason for the mHPA phenotype.

The article "Identified PAH V230A and PAH V230I mutations in a family with diverse clinical presentations" was published in 2024. Journal: Clin Case Rep.

## 2 CASE PRESENTATION

A 32‐year‐old woman was referred to the laboratory with her family to do a trio genetic test for her child, who was affected by PKU (Figure 1). Written informed constant statements were taken from all participants. This study was a part of our previous study, and it was approved by the Ethics Committee of Mashhad University of Medical Sciences.

**FIGURE 1:** Consanguineous family with a PKU member. (A) presents the Sanger's sequencing results of the affected child with PKU (V‐2), and her parents (III‐4 and IV‐8). (B) The pedigree of a consanguineous family with a PKU member.

Whole blood samples were taken from all three patients in EDTA tubes and DNA was extracted using the conventional salting out method. The quality and quantity of DNA were confirmed by nanodrop and gel electrophoresis. The disease‐causing variants were detected through step‐by‐step PCR amplification and sequencing of PAH gene exons. At first, the most common exons bearing mutations in Iranian patients (exons 6 and 7) were analyzed in the affected child (V‐2), and the results showed p.[V230A];[V230A] genotype. Then the affected exon was analyzed in both parents (IV‐8 and III‐3) to validate the genotype of V‐2. The III‐4 subject (father) was heterozygous for p.[V230A] mutation, and unexpectedly IV‐8 case (the mother) was bearing a compound heterozygous genotype (p.[V230A];[V230I]). The exon 6 was analyzed for IV‐8 subject using forward and reverse primers and the results confirmed the findings. The variants were described based on the sequence of NM_000277.3 transcript of the PAH gene, and following HGVS (Human Genome Variation Society) nomenclatures. The two mutations detected in this (c.689 T> C and c.688G> A respectively).

The level of serum Phe was measured in the subjects who had two mutations within the PAH gene (V‐2 and IV‐8 cases) in Akbar pediatrics hospital. Then the phenotype was classified based on the highest phenylalanine level: classic PKU (>1200 μmol/L), mild PKU (360–1200 μmol/L), and mHPA (120–360 μmol/L).^14^ The result of Phe assessment for IV‐8 case was higher than the normal range (179 μmol/L) which indicates mild hyperphenylalaninemia (mHPA) phenotype. She was conscious enough to raise up her three biological daughters and manage their lives as a housewife. However, she was not aware of her condition and never had taken any Phe‐free diet or Phe lowering medicine. The Phe concentration was assessed in V‐2 earlier and she presented mild PKU phenotype. The V‐2 case was not responsive to BH4 (taking a 24 and 48 h BH4 loading test).

The article "Identified PAH V230A and PAH V230I mutations in a family with diverse clinical presentations" was published in 2024. Journal: Clin Case Rep.

## 3 METHODS

The p. V230A and p. V230I (c.689 T > C and c.688G > A, respectively) variants were analyzed by various software programs (SIFT, PolyPhen‐2, CAAD, Mutation taster, and Mutation assessor) to predict the possible effect of amino acids substitution on the structure/function of PAH protein and assess the evolutionary conservation of the mutated region. The p.V230I was predicted to be tolerated, benign, likely benign, and neutral by most of the software (Table 1). However, the p.V230A variant was predicted to be deleterious, damaging, and disease causing by most of the prediction tools except CAAD which predicted it to be likely benign (Table 1). Both of mutations were reported to be likely pathogenic in ClinVar, yet only the V230I variant was reported in heterozygous state in population databases. Although p.V230A was not reported in population databases the pathogenicity score for p.V230A is generally higher than p.V230I.

**TABLE 1:** The results of p.V230I and p.V230A analysis using prediction tools and disease/population databases.

Variant	Prediction tools					Disease/population databases		
	SIFT	PolyPhen‐2	CAAD	Mutation taster	Mutation acessor	ClinVar	ExAC	1000 genome
p.V230I	Tolerated (0.29)	Benign (0.090)	Likely benign (18)	Disease causing	Neutral (0.9)	Likely pathogenic	Found in the heterozygous state	Found in the heterozygous state
p.V230A	Deleterious (0)	Probable damaging (0.989)	Likely benign (26)	Disease causing	Medium (0.887)	Likely pathogenic	Not found	Not found

The mutated PAH proteins bearing p. V230A and p. V230I variants were modeled via SwissModel online software according to the sequence of NM_000277.3 transcript of the PAH gene available at Ensemble. The crystal structure of the monomer form of the human PAH enzyme with PDB ID = 6HYC^15^ was selected as the most appropriate template because its blast result to the PAH protein reference sequence showed high coverage and identity. This primary model was used for further analysis of hydrogen bonds by the Swiss‐Pdb Viewer (version 4.1.0) visualization via Pymol software (version 1.1).

## 4 RESULTS

Protein modeling demonstrated alternations in the catalytic domain of the PAH enzyme. The substitution of Alanine, a non‐branched amino acid with Val 230, a small branched amino acid, can affect PAH structure more dramatically, in comparison to Isoleucine, another branched amino acid (Figure 2).

**FIGURE 2:** Presenting the result of protein modeling. (A) Visualization by PyMol. (B) H‐bonds analysis of mutated PAH proteins bearing p.V230I and p.V230A mutations in comparison with wild‐type PAH protein.

The article "Identified PAH V230A and PAH V230I mutations in a family with diverse clinical presentations" was published in 2024. Journal: Clin Case Rep.

Analysis of H‐bonds and comparing mutated proteins with wild type demonstrated an increase in H‐bonds length. The Val 230 residue created two H‐bonds with adjacent residues Leu 234 (2.89 Å) and Phe 233(3.26 Å). The p.V230I substitution results in the increase of H‐bond length to both Leu 234 (2.92 Å) and Phe 233(3.28 Å). The p.V230A variant increases the length of the H‐bond to Leu 234 (2.96 Å) as well. However, it has a more significant effect on the h‐bonds distance that the h‐bond between Val230 and Phe233 in wild‐type protein is clashed in p.V230A substitution (Figure 2).

## 5 DISCUSSION

Phenylketonuria, a hereditary defect of the PAH enzyme, might result in severe brain defects, following Phe accumulation. Therefore, early initiation of treatment can mainly prevent further injuries. However, current key treatment option, dietary management, has challenges and side effects if used in long term.^5^, ^6^, ^7^, ^8^ According to recently published guidelines patients with a specific range of serum Phe concentration do not need treatment.^1^ Thus, it is important to detect patients who can benefit from a life without medical intervention or dietary restriction at an early age.

In this study, a consanguineous family consisting of a PKU patient and her parents was analyzed for mutations within the PAH gene. The compound heterozygous genotype detected in one of the normal parents (case IV‐8) was approximately unexpected as she was conscious enough to manage her life and children and never had taken any Phe‐restricted diet during her lifetime (even in childhood or pregnancy). However, adults with HPA might be diagnosed in countries such as Iran where PKU newborn screening (NBS) started years after its development. Considering that PKU NBS implemented across Iran since 2012,^16^ the detection of such cases might be anticipated. Detecting a compound heterozygous genotype in the asymptomatic mother triggered further investigations of the Phe level. Evaluation of Phe level in case IV‐8 demonstrated a serum Phe level that was above the normal range and indicated mHPA phenotype (179 μmol/L). According to recent guidelines patients with untreated Phe concentration below 360 μmol/L, even women who are trying to conceive or are during pregnancy, do not need treatment.^17^ The IV‐8 case is an example that followed mentioned recommendation within whole her life even during the critical period of pregnancy inadvertently. As she was not aware of her condition and never had Phe restricted diet or taken intervention to lower the Phe level in her lifetime, she was considered to be an asymptomatic adult with mHPA. There have been reports of cases who progressed from mHPA to Phe level over 360 μmol/L, which is currently a borderline for the commence of treatment.^10^ Since the IV‐8 patient did not show PKU severe symptoms, she might always have stable Phe level <360 μmol/L which might be due to a specific genotype p.[V230I];[V230A]. Therefore, it was important to find out about the features of the mutations causing this phenotype and report them. Since genotype association with in vitro residual enzyme activity has been demonstrated for many PAH variants,^12^ prediction of phenotype based on genotype might be useful for genetic counseling and treatment recommendation.^13^

The article "Identified PAH V230A and PAH V230I mutations in a family with diverse clinical presentations" was published in 2024. Journal: Clin Case Rep.

The genotype and phenotype observed in V‐2 and IV‐8 were similar to reports in the BIOPKU database: p.[V230I];[V230A] genotype was reported to cause mHPA phenotype and p.[V2030A];[V230A] was observed with classic phenotype in the BIOPKU database.^18^ The allelic phenotype value (APV) for p.V230I is reported to be 10.^19^ APV is a value that shows the severity of a variant and its association with a corresponding phenotype.^19^ The p.V230I pathogenic variant showed the highest APV, which indicates the mildest HPA phenotype.^19^ According to genotypic phenotype values (GPVs) which are calculated as the APV with the highest value of the two APVs in a genotype, the metabolic phenotype is caused by the variant with higher PAH activity and APV, so this variant has the dominant role in determining phenotype.^19^ Additionally in a genotype compromising variants with unknown and 10 APV, the predicted phenotype will be mHPA^19^ as was observed in this study. Therefore p.V230I might be the main reason for this phenotype, as it retains 63% of enzyme activity and has caused mHPA phenotype in the homozygous state according to reports of BIOPKU.^18^ Comparison is not possible as APV and residual activity for p.V230A are unknown. However, p. V2030A has been reported to cause classic phenotype in the homozygous state (p.[V2030A];[V230A]) in BioPKU.^18^

The computational analysis demonstrated that both of the mutations are disease causing because they were detected only in heterozygous form in population databases (ExAC and 1000 genome) and were predicted to change protein function by prediction tools that used diverse algorithms. However, they cause different phenotypes. The variation in pathogenicity and subsequent phenotype might be underlined on affecting protein structure differently. Protein modeling demonstrated both mutations affected catalytic domain of the PAH enzyme but in different ways, so it might result in different enzyme activity subsequently. Protein modeling showed the p.V230I variant with high residual enzyme activity and APV has a less severe effect on H‐bonds in the same region in comparison with p.V230A which resulted in clash of one of the H‐bonds. These results confirmed phenotypic and other computational findings. Further functional studies are recommended to find more information about p. V2030A characteristics.

The article "Identified PAH V230A and PAH V230I mutations in a family with diverse clinical presentations" was published in 2024. Journal: Clin Case Rep.

## 6 CONCLUSION

In conclusion, it has a significant value to perform genetic testing and detect PKU patients who can benefit from a life without medical intervention or dietary restriction in early ages. This study presented the p. V230I pathogenic variant to be responsible for the mHPA phenotype which was detected in the asymptomatic adult and should be taken into account when considering genetic counseling and treatment for families with members harboring p.[V2030I];[V230A] genotype. In addition, further functional studies are recommended to gain a better understanding of the characteristics of p.V230A mutation and its impact on enzyme activity and PKU phenotypes.

## AUTHOR CONTRIBUTIONS

**Faeze Khaghani:** Conceptualization; investigation; methodology; software; visualization; writing – original draft; writing – review and editing. **Peyman Eshraghi:** Conceptualization; funding acquisition; investigation; resources; validation. **Tayebeh Hamzehloei:** Funding acquisition; resources; supervision; writing – review and editing.

## FUNDING INFORMATION

This study was funded by Mashhad University of Medical Sciences (MUMS), Iran. This study is part of Faeze Khaghani's MSc thesis.

## CONFLICT OF INTEREST STATEMENT

The authors declare that they have no conflict of interest.

## ETHICS STATEMENT

This study was a part of our previous study, and it was approved by the Ethics Committee of Mashhad University of Medical Sciences.

## CONSENT

Written informed consent was obtained from the patient to publish this report in accordance with the journal's patient consent policy.

## Data Availability

The data that support the findings of this study are available from the corresponding author upon reasonable request.

## References

[1] van Spronsen FJ , Blau N , Harding C , Burlina A , Longo N , Bosch AM . Phenylketonuria. Nat Rev Dis Prim. 2021;7(1):36.34017006 10.1038/s41572-021-00267-0PMC8591558

[2] De Groot M , Hoeksma M , Blau N , et al. Pathogenesis of cognitive dysfunction in phenylketonuria: review of hypotheses. Mol Genet Metab. 2010;99:S86‐S89.20123477 10.1016/j.ymgme.2009.10.016

[3] Sumaily KM , Mujamammi AH . Phenylketonuria: a new look at an old topic, advances in laboratory diagnosis, and therapeutic strategies. Int J Health Sci. 2017;11(5):63‐70.PMC566951329114196

The article "Identified PAH V230A and PAH V230I mutations in a family with diverse clinical presentations" was published in 2024. Journal: Clin Case Rep.

[4] Vardy ER , MacDonald A , Ford S , et al. Phenylketonuria, co‐morbidity, and ageing: a review. J Inherit Metab Dis. 2020;43(2):167‐178.31675115 10.1002/jimd.12186

[5] Crujeiras V , Aldámiz‐Echevarría L , Dalmau J , et al. Vitamin and mineral status in patients with hyperphenylalaninemia. Mol Genet Metab. 2015;115(4):145‐150.26123187 10.1016/j.ymgme.2015.06.010

[6] Enns G , Koch R , Brumm V , et al. Suboptimal outcomes in patients with PKU treated early with diet alone: revisiting the evidence. Mol Genet Metab. 2010;101(2–3):99‐109.20678948 10.1016/j.ymgme.2010.05.017

[7] Evans S , Daly A , MacDonald J , et al. The micronutrient status of patients with phenylketonuria on dietary treatment: an ongoing challenge. Ann Nutr Metab. 2014;65(1):42‐48.25196394 10.1159/000363391

[8] Van Wegberg A , Macdonald A , Ahring K , et al. The complete European guidelines on phenylketonuria: diagnosis and treatment. Orphanet J Rare Dis. 2017;12(1):1‐56.29025426 10.1186/s13023-017-0685-2PMC5639803

[9] Blau N , van Spronsen FJ , Levy HL . Phenylketonuria. Lancet. 2010;376(9750):1417‐1427.20971365 10.1016/S0140-6736(10)60961-0

[10] Berlin CM Jr , Levy HL , Hanley WB . Delayed increase in blood phenylalanine concentration in phenylketonuric children initially classified as mild hyperphenylalaninemia. Screening. 1995;4(1):35‐39.

[11] Viall S , Ayyub O , Rasberry M , Lyons K , Ah Mew N . "mild" hyperphenylalaninemia? A case series of seven treated patients following newborn screening. Mol Genet Metab. 2017;122(4):153‐155.29102225 10.1016/j.ymgme.2017.10.010

[12] Himmelreich N , Shen N , Okun JG , Thiel C , Hoffmann GF , Blau N . Relationship between genotype, phenylalanine hydroxylase expression and in vitro activity and metabolic phenotype in phenylketonuria. Mol Genet Metab. 2018;125(1–2):86‐95.30037505 10.1016/j.ymgme.2018.06.011

[13] Hillert A , Anikster Y , Belanger‐Quintana A , et al. The genetic landscape and epidemiology of phenylketonuria. Am J Hum Genet. 2020;107(2):234‐250.32668217 10.1016/j.ajhg.2020.06.006PMC7413859

[14] Schiff M , Sarafoglou K , Hoffmann GF , Roth KS . Pediatric endocrinology and inborn errors of metabolism. J Inherit Metab Dis. 2017;40(6):893.

[15] Flydal MI , Alcorlo‐Pagés M , Johannessen FG , et al. Structure of full‐length human phenylalanine hydroxylase in complex with tetrahydrobiopterin. Proc Natl Acad Sci. 2019;116(23):11229‐11234.31118288 10.1073/pnas.1902639116PMC6561269

[16] Davarani ER , Takaloo FM , Daneshi S , et al. Assessing the phenylketonuria (PKU) neonatal screening program and the incidence rates of PKU in Kerman County, Iran: a health system research. J Pediatric Neonatal Individ Med. 2022;11(2):e110217.

The article "Identified PAH V230A and PAH V230I mutations in a family with diverse clinical presentations" was published in 2024. Journal: Clin Case Rep.

[17] Van Spronsen FJ , van Wegberg AM , Ahring K , et al. Key European guidelines for the diagnosis and management of patients with phenylketonuria. Lancet Diabetes Endocrinol. 2017;5(9):743‐756.28082082 10.1016/S2213-8587(16)30320-5

[18] BIOPKU. http://www.biopku.org

[19] Garbade SF , Shen N , Himmelreich N , et al. Allelic phenotype values: a model for genotype‐based phenotype prediction in phenylketonuria. Genet Med. 2019;21(3):580‐590.29997390 10.1038/s41436-018-0081-x

